# Cold Chain Management by Healthcare Providers at a District in Ghana: A Mixed Methods Study

**DOI:** 10.1155/2021/7559984

**Published:** 2021-09-13

**Authors:** Anthoniette Asamoah, Nancy Innocentia Ebu Enyan, Abigail Kusi-Amponsah Diji, Charles Domfeh

**Affiliations:** ^1^Fomena Nursing and Midwifery Training College, Fomena, Ashanti Region, Ghana; ^2^Department of Adult Health, School of Nursing and Midwifery, University of Cape Coast, Cape Coast, Ghana; ^3^Department of Nursing, Kwame Nkrumah University of Science and Technology, Kumasi, Ghana; ^4^Department of Health, Physical Education and Recreation, University of Cape Coast, Cape Coast, Ghana

## Abstract

**Background:**

Despite the relevance of cold chain management in maintaining the potency of vaccines, gaps still exist in the ability of healthcare practitioners to maintain the cold chain system effectively. Thus, the current study sought to assess healthcare providers' knowledge, attitudes, practices, and challenges regarding cold chain management.

**Methods:**

A concurrent mixed methods study was conducted at twelve facilities in the Sekyere Central District of Ghana. Eighty-six (86) participants took part in a survey that assessed their “cold chain management” knowledge and attitudes. Twelve (12) cold chain sites within the district were also observed in respect of their cold chain management practices. Eleven key informants were additionally interviewed to explore their challenges on cold chain management. Quantitative data were analyzed using descriptive (frequencies, percentages, means, standard deviations, ranges) and inferential statistics (Spearman's rho correlation). Qualitative data were inductively analyzed into themes which described participants' challenges on cold chain management.

**Results:**

Majority of the participants scored ≥70% on knowledge (68.6%) and attitudes (67.4%) toward cold chain management. However, there was a very weak positive and statistically insignificant relationship between participant's knowledge and attitudes toward cold chain management (*r* = 0.109, *p* = 0.317). Regarding cold chain management practices, majority of the facilities had their vaccine vial monitors attached to the vaccines (8/12, 66.7%), had functional fridge tags (8/12, 66.7%), and an appropriate refrigerator to store vaccines (7/12, 58.3%). However, the study observed that 91.7% (11/12) of the facilities did not have policies and guidelines on cold chain management while all 12 facilities (100%) did not have a contingency plan in place for equipment. With regards to the cold chain management challenges, participants raised concerns about inadequate personnel, erratic power supply, logistical constraints, and transportation difficulties.

**Conclusion:**

Although majority of the participants had good knowledge and attitude towards cold chain management, there was a weak association between them. This implies that good knowledge may not necessarily influence good attitudes towards cold chain management and vice versa. The extent to which facilities support cold chain management practices was suboptimal. Participants encountered a number of challenges which prevented them from managing the vaccine cold chain system effectively. We recommend continual professional education for cold chain practitioners, provision of adequate human and material resources for cold chain management, and enhanced monitoring and evaluation of cold chain activities. Future studies should quantitatively measure individual participants' knowledge, attitudes, practices, and challenges on cold chain management so that we can establish the relationships that exist between these components.

## 1. Introduction

The achievement of higher vaccination coverage depends on the competent distribution of cost-effective vaccines that can be stored at the appropriate temperatures through quality cold chain management systems. Thus, effective cold chain management systems are critical in preserving vaccines from production to vaccination sites [1, 2]. Vaccines as biological medical preparations can easily lose their potency when they are not stored at the optimal temperature of +2°C to +8°C [2–4]. As part of measures to ensure the potency of vaccines, a standardized cold chain system consisting of efficient and reliable equipment, trained staff, and distribution of vaccines is required [5]. The importance of the efficient cold chain management system cannot be overemphasized as it prevents avoidable vaccine wastage which ultimately affects vaccine safety and vaccination coverage [6, 7].

Despite the training given to healthcare providers (HPs), evidence suggests that gaps in knowledge, attitudes, skills, and nonadherence to cold chain management practices negatively affect the efficient management of the cold chain system [8, 9]. These nonadherent attitudes and practices coupled with inadequate knowledge could break the cold chain management system and affect the quality of the vaccines that are to be administered to the populace. Additionally, vaccine safety may be compromised and result in vaccine-related morbidity and mortality, especially in vulnerable groups (children under 59 months and pregnant women). Furthermore, poor cold chain management creates financial difficulties and can serve as burden on the economy [10].

Although the Ghana Health Service's Expanded Programme on Immunization (EPI) is responsible for cold chain activities in Ghana, there is paucity of evidence on healthcare providers' knowledge, attitudes, and challenges on cold chain management as well as the extent to which health facilities adhere to cold chain management in Ghana [8, 11–13]. The Ministry of Health in collaboration with the Ghana Health Service has also developed a guideline on vaccination which includes the cold chain management system [7]. By virtue of the identified research gaps and as part of the efforts to assess the extent of adherence to existing guidelines, the current study sought to assess healthcare providers' level of knowledge, attitudes, practices, and challenges on cold chain management.

## 2. Methods

### 2.1. Study Design and Setting

A concurrent mixed methods study design was used; quantitative and qualitative design approaches were deemed appropriate in answering different research questions.

The study was conducted at the Sekyere Central District which is one of the thirty (30) administrative districts, located in the northern part of the Ashanti Region. It shares boundaries with Mampong Municipal, Atebubu, Sekyere East, Sekyere South, and Ejura-Sekyere Odumasi districts. The district has been subdivided into five subdistricts (Nsuta, Kwamang, Birem, Oku and Asubuasu) with 150 communities, majority (70%) of which are in rural areas [14]. Additionally, the district has a couple of health centers and Community-based Health Planning and Service (CHPS) zones. It also has a disease control unit which oversees the implementation of the Expanded Programme on Immunization activities, disease surveillance, and the prevention of communicable diseases (District Health [15]). The total population of the district based on the 2010 census is 71,232. The population has a sex ratio of 49.5 for males and 50.5 for females. The total fertility rate for the district is 4.0. The crude death rate for the district is 7.65 per 1000 people. The district has a household population of 71,232 with a total of 4,902 households [14].

### 2.2. Study Population and Sampling

For the quantitative aspect of the study, the study population comprised of 129 healthcare providers aged 24 to 59 years who were working in the Sekyere Central District (District Health [15]). Participants were eligible for inclusion in the study provided they were working in a cold chain site during the period of the study. Participants who were on any type of leave (maternity, casual, study) during the study period were excluded.

The census sampling method was used as the researchers had sufficient resources to conduct the study among the targeted population. Out of the 129 healthcare providers, 23 were on leave during the study period for various reasons such as study purposes (*n* = 14), childbirth (*n* = 6), and other duties (*n* = 3). Of the 106 healthcare providers who were at post, 20 refused participation in the study due to the busy nature of their work schedules. This resulted in a response rate of 81.1%.

For the qualitative component of the study, purposive, and maximum variation (with a focus on age, gender, educational qualification, specialty, working experience, and geographical location), sampling techniques were used in selecting 11 healthcare providers who served as key informants for the individual face-to-face interviews. This was supported by Creswell's recommendation of attaining data saturation with 5-25 participants [16].

### 2.3. Data Collection Procedure

Two research assistants were recruited and trained to assist with the data collection following administrative and ethical approvals. An initial contact was made with the District Director of Health Services who introduced the principal investigator and research assistants to the Facility and Unit Heads. Afterwards, the investigators approached the potential participants and informed them about the study aim and procedures before giving their verbal and written consent. In order to ease the response burden on participants, the research assistants guided the participants by reading the items for their responses. On average, about 30 minutes was spent by participants in answering the questionnaires.

A day was spent at each of the 12 cold chain sites to assess the extent to which the facility supported cold chain management practices. With the assistance of an observational guide and the Unit Heads in-charge of the vaccine cold chain systems, each of the outlined items was assessed and documented accordingly.

Key informant face-to-face individual interviews were conducted to explore their challenges on cold chain management. Each interview session took approximately 30-45 minutes and occurred at a convenient place and time for both parties. After obtaining participants' permissions, the interviews were audio recorded and transcribed verbatim.

### 2.4. Data Collection Instruments and Measurement

Three (3) data collection instruments were used in the study: a structured questionnaire, an observational guide, and a semistructured interview guide. These instruments were developed based on existing literature [17–22] and policy guidelines on immunization in Ghana [7].

### 2.5. Structured Questionnaire

Participants' knowledge and attitudes on cold chain management were measured using a structured questionnaire. The questionnaire focused on the three subdomains: participants' background characteristics, their cold chain management knowledge, and attitudes. The background characteristics of the participants included the following: subdistrict, current place of work, category of staff, age, gender, educational qualification, working years in general, years of experience in cold chain management, and years spent in vaccine administration. In the context of our study, “knowledge” was defined as the information and understanding of participants regarding cold chain management; “Attitudes” also referred to the healthcare provider's level of commitment to cold chain management practices.

Participants' knowledge and attitudes were assessed on cold chain management issues such as vaccine handling and transportation, storage, vial monitoring, multidose vial policy, freeze-sensitive vaccines, and their assessment. The “knowledge” subdomain consisted of 20 items, of which participants were required to respond by answering “Yes” or “No.” Correctly indicated knowledge items were rated as one (1), whereas incorrect responses were given a score of zero (0). Thus, the maximum attainable score on knowledge was 20. Participants' knowledge scores were converted into percentages using the formula: (score obtained/20) × 100. Consistent with earlier studies [18, 19], the “knowledge scores” were categorized as follows: poor (0-50%), fair (51-69%), and good (≥70%).

The “attitude” subdomain also comprised of 10 statements which required participants to indicate their level of agreement or disagreement on a Likert-scaled options from 1 to 5, where “1,” “2,” “3,” “4,” and “5” corresponded with “strongly disagree,” “disagree,” “neutral,” “agree,” and “strongly agree,” respectively. Both positive and negative statements were constructed to control response bias. Statements which required the participant to “agree” or “strongly agree” were recoded and given a score of one (1). All other responses to such statements (“neutral”, “disagree” or “strongly disagree”) were restructured and rated as zero (0). Alternatively, negative worded “attitude” statements were reversely coded and scored. The highest attainable score on “attitude” was 10, and scores obtained by participants were translated into percentages using the formula: (obtained score/10) × 100. In line with previous literature [18, 19, 21], the “attitude” scores were classified as poor (0-50%), fair (51-69%), and good (≥70%).

### 2.6. Observational Guide

The extent to which each of the 12 included facilities supported cold chain management practices was assessed using a structured observational guide. The guide consisted of 49 items which were further grouped into three subdomains: “policies, procedures and guidelines” (14 items), “quality of vaccine care” (22 items), and “equipment” (13 items). The presence or absence of items outlined in the guide was noted at each cold chain site. Furthermore, the number of facilities which had or did not have a particular item was compiled and presented as frequencies and percentages.

### 2.7. Interview Guide

With the aid of a semistructured interview guide, the challenges of cold chain management were explored. In the present study, “challenges” were defined as the internal or external factors that prevented a healthcare provider from achieving expected cold chain management system outcomes.

### 2.8. Validity, Reliability, and Trustworthiness

Validity and reliability of the quantitative data collection instruments (questionnaire and observational guide) were assessed. Face and content validity of the structured questionnaire and observational guide were determined by three experts in the fields of Public Health and Nursing before its use in the current study. The validated questionnaires were subsequently pretested with forty (40) healthcare providers at four similar facilities with the aim of assessing the instruments' internal consistency. The Kuder Richardson (KR20) reliability coefficient was used in the assessment of the instrument's internal consistency as there was a correct answer for each item on the “knowledge,” recoded “attitude” subdomains as well as the observational guide that measured the extent to which the four facilities supported cold chain management practices. The reliability coefficient for the 20-item “knowledge” subdomain was 0.761, and that of the 10-item “attitude” subdomain was 0.723, whereas that of the extent to which the four facilities supported cold chain management practices was 0.742. These reliability coefficients signified an acceptable level of internal consistency of the instruments.

The researchers employed several strategies to enhance trustworthiness in the qualitative component of the study which used individual interviews to explore participants' challenges on cold chain management. Adherence to Guba and Lincoln's [23] credibility, dependability, confirmability, and transferability was done to ensure trustworthiness. The use of the same semistructured interview guide, verbatim transcription of audio-recorded interviews, member checking, coding by two researchers, and consensus building on the actively generated themes enhanced credibility. The process of comparing and contrasting the codes and themes generated by each of the four researchers also promoted the confirmability and dependability of the study findings. The thorough description of the research methods, processes, and findings enriched the study's transferability.

### 2.9. Data Analysis

The quantitative data were analyzed with the Statistical Product and Service Solutions (SPSS) version 20.0. Continuous variables were presented using means, standard deviations, and ranges (minimum–maximum). Categorical variables were illustrated as frequencies and percentages. The relationship between participants' cold chain management “knowledge” and their “attitudes” was examined using Spearman's rho correlation analysis as we were dealing with two ranked variables.

Inductive analyses of the qualitative interviews were manually done. The basic unit of meaning (codes) was initially generated before merging them into themes which described participants challenges on cold chain management. The entire process of thematic analysis was done by two members of the research team and comprised of six phases: familiarizing with the data, generating initial codes, searching for themes, reviewing the themes, and redefining and naming theme [24].

### 2.10. Ethical Considerations

Ethical approval with reference number UCCIRB/CES/2019/01 was obtained from the Institutional Review Board of University of Cape Coast in Ghana following administrative approval from the District Directorate. Ethical principles such as informed consent, confidentiality, autonomy, privacy, and voluntary participation were adhered to throughout the entire process of the research. Soft copies of participants' data were stored on a password protected pen drive, whereas the hard copies were kept in a locked cabinet located in the principal investigator's office and accessible only to the researchers involved in the study.

## 3. Results

### 3.1. Sociodemographic Characteristics of the Participants Involved in the Survey

As illustrated in Table 1, majority of the participants were aged 26–30 years (55.8%) with a mean of 30 years and standard deviation of 4 years. Majority of them were females (60.5%) and had obtained “certificate” as their highest level of educational qualification. Slightly over half of the participants were community health nurses (52.4%); over 40% of the participants were also from the Nsuta subdistrict. More than half of the participants had spent less than five years working in the Ghana Health Service (52.3%), cold chain management (61.6%), and vaccine administration (61.6%).

### 3.2. Level of Knowledge and Attitudes of Healthcare Providers towards Cold Chain Management

Over two-thirds of the participants had good knowledge (68.6%) and attitudes (67.4%) regarding cold chain management (refer to Table 2). Results of Spearman's rho correlation analysis revealed a very weak, positive, and statistically insignificant correlation between knowledge and attitudes towards cold chain management (*r* = 0.109, *p* = .317).

### 3.3. The Extent to which Facilities Support Cold Chain Management

As illustrated in Table 3, eight out of the 12 facilities (66.7%) had the vaccine vial monitors (VVM) attached to all the vaccines in the refrigerator irrespective of the type of vaccine, and not just some few ones; that is, the VVM was clearly fixed (visible in line with manufacturers standard) on all the vaccines in the refrigerator irrespective of the type of vaccine so that the stage of VVM can be determined indicating the vaccine was in good condition. But for some of the facilities, the VVM attached to all the vaccines or a cluster of vaccines were not readable because it was fully or partially removed from the vaccine vails; so, the stage of the VVM reading could not be determined, this was due to the fact that the ice in the refrigerator was melting, the facilities do not have another source of power to fuel the refrigerator, or the refrigerator has technical challenges. VVM is expected to be fully fixed to the vaccine vail without any alteration so that the degree of heat sensitivity can be indicated. Good condition was assessed based on the presence of workable VVM on all vaccine vails irrespective of the type of vaccine or the quantity of vaccine in the refrigerator so that the state of the vaccine can be known to determine whether the vaccine is in good condition or not. Eight of the facilities also had functional fridge tags (66.7%), and seven facilities had an appropriate refrigerator to store vaccines (58.3%). However, the study observed that 91.7% of the facilities (11/12) did not have policies and guidelines on cold chain management. Additionally, the study found out that all the 12 facilities (100%) observed did not have a contingency plan in place for equipment.

### 3.4. Description of Participants Involved in the Key Informant Interviews

Three of the key informants were recruited from Nsuta subdistricts while two each were selected from Kwamang, Birem, Oku, and Asubuasu subdistricts. Key informants consisted of two public health officers, one field technician, and eight community health nurses. Two of the key informants were females while the other nine were males. Two were degree holders whilst the rest of the nine were certificate holders. The informants had a minimum age of 25 years and a maximum age of 35 years. The study found out that three of the participants had spent less than five years in the Ghana Health Service, six had spent between five to 10 years, and two had spent 11 to 15 years. Seven of them had spent less than five years in cold chain management whilst the remaining four had spent five to 10 years in cold chain management. Six had less than five years' experience in vaccine administration, and five had served for five to 10 years in vaccine administration.

### 3.5. Exploration of the Challenges on Cold Chain Management

Inductive analysis of the interview data revealed three themes which described the cold chain management challenges. These were “state of constant pressure and stress,” “irregularities in the maintenance of vaccine temperatures,” and “delays in reaching the underserved communities.”

### 3.6. State of Constant Pressure and Stress

This theme denotes the continuous pressures that were constantly placed on the participants due to their lack of control on external factors such as personnel and power supply. Participants reported insufficient staff who have been adequately trained on the cold chain management system. This subsequently led to constraints as they have to work beyond their working schedules in their pursuit of maintaining the vaccine cold chain systems and serving their assigned communities. While participants reported of the absence of power supply in some districts, others lamented about the unreliable nature of their available power supply. Additionally, most of the facilities with a power source also relied heavily on electrical energy (electricity) with few using solar energy. Those facilities that were using electrical energy (electricity) complained about the facility's inability to acquire power supply back-ups such as solar, generator, or plant. By virtue of the unreliable power source, participants reported of constantly being under pressure and stressed as they had to be constantly prepared for any unforeseen factors which were beyond their control. The following excerpts support this theme:

*The community health nurses here are five but two (2) are managing it. No is not enough because we can be transferred or we can travel so it would be better if we would be all trained about the cold chain system so that everybody can get access to it if one is not there the other person can handle it. (CCA).*

*With the main three that I gave I would sideline electricity challenge that we have been having at the facility whenever there are outrages the facility is also not having a plant or generator that can support the facility with electricity so that we can maintain our cold chain system as expected of us that is the main challenge that we have at the facility now* (CCC).

### 3.7. Irregularities in the Maintenance of Vaccine Temperatures

This theme illustrates the logistical constraints and healthcare malpractices that threatened the temperature regulation of vaccines. According to the participants, the facilities did not have sufficient supply of cold chain logistics such as refrigerators, cold boxes, and vaccine carriers. The insufficient cold chain logistics were sometimes deficient in their functioning and needed repair or replacement as some of them had outlived their period of optimal performance. Some of the participants also admitted to having challenges in handling the digital fridge tag device as the use of thermometers were phasing out of the system. In subdistricts where the thermometers were still in use, they reported of their nonfunctioning nature which created difficulties in regulating vaccine temperatures and resulted in the frequent opening of the fridge for temperature assessment purposes. As a result of these logistical constraints, the vaccines were sometimes stored below the minimum temperature range of 2°C or above the maximum recommended temperature of 8°C. One of the participants had this to say:

*Even if you go to Nsuta subdistrict which is the, should I say the subdistrict capital even vaccine carriers they do not have, the vaccine carriers are broken, some of them do not have foams,… in fact some of the carriers are not in good shape. I talked about the vaccine fridges… the carriers and even the cold boxes we do not have adequate numbers… this vaccine fridge that is sitting here is not functioning properly. The slightest mistake, all your vaccines would get frozen so that one too is a challenge, we still have the RCW50 vaccine fridges in the system, which excuse me for the want of a better word, obsolete because the parts are not on the market* (CCD).

Participants also reported of some attitudes and behaviors which had the potential of altering the recommended temperatures for the storage of vaccines. Some of these attitudes and behaviors included the placement of drinks and water in the vaccine refrigerators which led to its frequent opening, potentially exposing the temperature-sensitive vaccines to heat. Other undesirable behaviors reported by participants included the inappropriate placement of the fridge tags, improper chatting of the temperature, and removal of the vaccine vial monitors which creates difficulties in ascertaining the potency of vaccines. One participant recounted these behaviors as follows:

*The thing is the fridge is a vaccine fridge and we are supposed to put only vaccines into the fridge, not any other thing so as you are putting water and drinks into it, it would lead to frequent opening of the fridge and this can bring heat into the fridge and it would spoil the potency of the vaccine okay we do that* (CCB).

### 3.8. Delays in Reaching the Underserved Community

This theme described the transportation challenges participants faced in getting potent vaccines from their source to the targeted community or users. Due to the nonavailability and nonfunctioning nature of some cold chain logistics (such as refrigerators, cold boxes, and vaccine carriers), HCPs have to travel long distances to other facilities to pick up vaccines which has cost implications and also delay the time that they have to reach the communities they serve. Also, due to the unreliable power supply at most subdistricts, some HCPs have to travel to far distances to get ice packs for their vaccines which creates inconveniences in their planned vaccination schedules and sometimes affect the vaccine's potency. Participants reported of poor transportations systems within some parts of the district which affected their ability to get access to icepacks at designated places to keep the vaccines at the recommended temperature ranges. Participants further reported of the inconveniences of travelling long distances from their place of residence to the workplaces several times to check on the state of the vaccines outside their working schedule due to the unreliable nature of the power supply systems. Some participants had this to say:

*“You have to ride a motorbike to a far distance to get ice packs for our vaccines … they keep their vaccines at Nokwareasa CHPS compound so they have to commute to Nokwareasa to take vaccines every day because sometimes you have to bring some of the vaccines to the facility for the next day outreach activities because we don't have a fridge”* (CCE).

*“When you have light off throughout the whole of a week or three days is a challenge for the management of cold chain in this facility and then one time too again weekends is another challenge for me; where I reside from that place to here to me is a challenge sometimes you have to go evening, morning and those kinds of things so is another challenge”* (CCF).

## 4. Discussion

The current study is aimed at assessing healthcare providers' knowledge, attitudes, practices, and challenges regarding cold chain management. The study revealed that majority of the participants had good knowledge and attitudes towards cold chain management. Nevertheless, there was a weak positive association between participants' knowledge and attitude. This shows that knowledge may not always influence practitioners' attitude on cold chain management in reality and vice versa. A significant proportion of the facilities did not have policies to guide the management of cold chain which resulted in suboptimal practices within the district. The healthcare providers also narrated a myriad of resource (human and material) challenges which impeded the effective management of the cold chain system in the district. Detailed discussions of the study findings have been provided below.

### 4.1. The Level of Knowledge of Healthcare Providers on Cold Chain Management

The study assessed the level of knowledge of health practitioners on cold chain management. The findings suggest that about two-thirds of the health practitioners had a good level of knowledge on cold chain management (68.6%). A possible explanation of this could be that the district organized a refresher training for a section of the staff on cold chain management as part of a supplemental immunization activity (SIA) that took place in the country in 2018. Again, majority of the participants were community health nurses who constantly work with vaccines or are involved in aspects of cold chain management. Earlier studies also reported high knowledge of the respondents on cold chain management [17, 25–27]. However, the knowledge was slightly higher compared to the current study. The differences in settings and some other contextual factors including access to materials and information could influence the outcome of these studies. For instance, Azira's study was conducted in Malaysia where there may be well-developed infrastructure for cold chain management, as compared to the current study that was conducted in a district where some of the facilities do not have access to the internet or policy guidelines on cold chain management [17]. Although two-thirds of the participants had a good knowledge of cold chain management, the remaining one-third who had poor and fair knowledge is a cause for concern. This calls for sustained educational efforts to enhance health practitioners' knowledge as similar knowledge gaps have been raised by Diamenu and colleagues [12] on cold chain management in Ghana. This is an important area to address as a high level of knowledge among health practitioners directly working with vaccines that is critical in ensuring the potency and safety of vaccines and effective maintenance of the cold chain system [28].

### 4.2. The Attitude of Healthcare Providers towards Cold Chain Management

The attitudes of health professionals working with vaccines are vital to the achievement or failure of vaccination programmes [29]. Two-thirds of the healthcare providers in the current study had good attitudes toward cold chain management. A plausible explanation could be that the participants may have responded to the attitude component of the questionnaire in a way that put them in good light due to the self-reported nature of this component. The attitude seems to be an important health behavior concept which could lead to the achievement of desirable behavior. Therefore, a high proportion of the participants demonstrating a good attitude may facilitate effective management of the cold chain system.

Previous studies have reported positive attitudes towards cold chain management [1, 18, 21]. A plausible explanation is that a positive attitude may influence the practice of maintaining vaccine cold chain management systems [30]. Nonetheless, the findings of the current study are inconsistent with that of Azira and colleagues [17] in which the participants had poor attitudes towards cold chain management. The inconsistencies could be due to the differences in the sociodemographic backgrounds of the participants and the context within which the studies were conducted. Additionally, differences in the level of supervision, leadership, policy implementation, and the facilities available to support health practitioner's effective management of cold chain could be attributable to the observed differences.

### 4.3. Relationship between Knowledge and Attitude of Healthcare Providers regarding Cold Chain Management

It is worth mentioning that though more than half of the healthcare providers had good knowledge and attitudes towards cold chain management, the relationship between knowledge and attitudes was found to be weak. This implies that good knowledge of cold chain management may not necessarily lead to positive attitudes towards cold chain management in the studied participants and vice versa. Contrary, a study conducted in Nigeria reported positive attitudes despite gaps in knowledge of cold chain management [2]. Differences in the setting and other contextual issues might explain the observed findings.

### 4.4. The Practice of Cold Chain Management

The extent to which facilities support cold chain management is important in assuring the public of the safety and potency of vaccines. The management of vaccines does not depend on infrastructure alone, but adherence to best practices and standards for effective management of the cold chain system [17]. Findings of this study indicated that the majority of the facilities had their vaccines in good condition as confirmed by the state of the vaccine vial monitors (VVMs) that were attached to all the vaccines stored in the refrigerators. Even though these findings were reassuring, there is also cause for concern as the VVMs were not attached to all the vaccines. This is worrying as there may be some vaccines with questionable VVM status in the district which may have implications for public health safety when used during vaccinations.

It is also worth mentioning that most of the facilities had functional fridge tags while others were not in possession of a refrigerator in the first instance. The availability of fridge tags aids in temperature monitoring of the vaccines in the refrigerator. Thus, the absence of fridge tags implies that some cold chain sites are not effectively monitoring the vaccine temperatures within the refrigerators. Considering the sensitivity of vaccines to temperature fluctuations, this raises concerns about the vaccine management and its proper storage for use in public health activities. Also, the absence of refrigerators in some facilities has dire implications on vaccine health as vaccines are more likely to be stored under suboptimal conditions and may ultimately affect the ability of vaccine to prevent diseases.

Preferably, all cold chain refrigerators at the district level are to maintain a temperature of +2°C to +8°C as the optimal temperature range for the storage of vaccines at the district and subdistrict level [5]. Accidental freezing can cause damage to freezing sensitive vaccines such as diphtheria, pertussis, tetanus, Hemophilus influenza type B, and hepatitis B (DPT/ HIB/HEP) [5]. A previous study reported that most of the health facilities had at least one ice-lined refrigerator, a deep freezer, and functional thermometers that aided in the management of the vaccine cold chain [19]. In Ghana, the capacity of cold chain activities at the national level seems to be adequate for both positive and negative storage but there is a disparity at the regional and district levels which is basically due to inadequate cold chain storage capacity [31].

Consistent with a previous study [2], many of the facilities did not have policies and guidelines on cold chain management practices. The importance of protocols and guidelines on cold chain management especially in remote areas with poor telecommunication network cannot be overstated as they serve as useful guides in the effective management of vaccine cold chain systems. Furthermore, the study found out that all the 12 facilities observed did not have a contingency plan in place for equipment. Meanwhile, a contingency plan helps facilities to identify resources to put in measures to curtail risk [32]. This practice is expected to be applied in all health facilities that are handling the vaccine cold chain system. Consequently, in case of a breakdown of the cold chain system, there is the possibility that volumes of vaccines could be wasted due to a lack of preparedness.

### 4.5. Exploration of the Challenges to Cold Chain Management

Participants described a host of challenges which were themed as follows “state of constant pressure and stress,” “irregularities in temperature maintenance,” and “delays in reaching the underserved communities.” Discussion of these themes has been provided below.

### 4.6. State of Constant Pressure and Stress

The findings suggested a “state of pressure” that were experienced by healthcare providers due to their lack of control on external factors such as power supply and logistical constraints. A possible explanation is that some of the facilities lack access to electricity or source of power such as gas or kerosene. This challenge could potentially lead to poor performance and may affect the vaccine cold chain and herd immunity. For instance, refrigerators that depend on electrical power will not be operational within such areas, which could have a lot of consequences on vaccination, especially among vulnerable groups (children under 59 months and pregnant women). Additionally, some health professionals in an attempt to innovate alternative strategies may end up storing vaccines under inappropriate conditions. This finding corroborates with that of an earlier study which reported that in some countries, vaccines may be exposed to heat and frozen temperatures, especially when transported to remote areas [33]. These practices ultimately affect the potency and safety of vaccines.

The problem of erratic power fluctuations that emerged in this study has also been reported in previous studies [1, 34]. Ateudjieu and colleagues [34] indicated that only 7 facilities out of 34 had access to a permanent power supply. Power outages could lead to changes in temperature which can affect the molecular nature of the vaccines. The longer the duration of the power fluctuation, the higher the chances of the vaccines losing their potency. Power fluctuations can also destroy certain refrigerators depending upon their capacity to stabilize power flow. These circumstances can result in the destruction of large volumes of vaccine, especially the heat-sensitive ones. Dissimilar to the present study findings, earlier studies by Ateudjieu et al. [34] and Ogboghodo et al. [1] reported that most of their facilities had access to a power supply which could facilitate effective management of the vaccine cold chain.

The study also found out that inadequate equipment was a contributing factor to the challenges of cold chain management. If cold chain equipment is not available, vaccines are going to be destroyed, and the targeted populations may be at risk of being vaccinated with inefficacious vaccines. This was reported by Timóteo et al. [35], and a similar finding was also reported by Ateudjieu et al. [34]. Although there were methodological variations between these studies and the current study, equipment inadequacy is still a challenge to today's cold chain management. Our findings are also affirmed by Bogale, Amhare, and Bogale [9] who reported that some of the facilities lacked refrigerators.

In the same way, it was observed that the facilities involved in the current study lacked an alternative source of power or energy. This finding is not consistent with that reported by Yassin et al. [27] as most of their facilities had available power source (generator/solar). In a related study, the facilities had backup gas bottles to support cold chain management in case of power failure [36]. Meanwhile, it is expected that facilities that store vaccines get a standby generator or an alternative power supply. With this situation, facilities may be tempted to buy “ice block” to store the vaccines, especially, during long outreach hours. These ice blocks tend to dissolve the vaccine vial monitor (VVM) of the vaccines, peel them off, which makes VVM reading either difficult or impossible.

Furthermore, poor maintenance of faulty equipment also emerged as a challenge. However, equipment is the pivot of cold chain management, and they need to be maintained as quickly as possible so that the vaccine cold chain would not be disrupted. When maintenance is delayed, vaccine potency is negatively affected, and this could lead to vaccine-induced/derived diseases and outbreaks when received by end-users [37].

### 4.7. Irregularities in Temperature Maintenance

Temperature maintenance is critical for effective management of the cold chain. This is because the potency of vaccines is attained through a certain optimal temperature range, where any alteration in temperature would render the vaccines inactive [38]. Contrary to a recent study [27] where most of the facilities recorded the temperature twice daily, the current study observed irregular charting of the temperature of the refrigerators. This finding indicates that faults cannot be detected on time, especially when outreaches have ceased at the end of the month. Also, when vaccines are not monitored, wastage could result due to poor contact with the refrigerator, since any rise in temperature or decrease in temperature is likely to affect one type of vaccine or the other as a result of their sensitivity to temperature discrepancies. Consequently, the optimal temperature of +2°C to +8°C or−20°C which needs to be maintained through appropriate monitoring and temperature regulation [39] is not achieved.

In line with earlier studies [2, 3, 40, 41], the current study observed the storage of other medications in the vaccine refrigerators. The introduction of other medications into the refrigerator introduces heat into the fridge since this affects the regulation of the temperature of the fridge. There is also the possibility of the other medications contaminating the vaccines by gradually leaving their residue in the fridge. Their aroma can also diffuse into the vaccines, adding up to the contamination process.

### 4.8. Delays in Reaching the Underserved Communities

Consistent with an earlier study [42], our study found that the participants were challenged with transportation issues. Health facilities with inadequate cold chain logistics often depend on other facilities for the needed assistance, which may interfere with vaccination activities. This situation forces some health professionals to keep vaccines in carriers for more than a day without changing icepacks. Furthermore, diluents, on the other hand, would not be stored a day before vaccination and could be reconstituted which can also cause thermoshock to vaccines. This calls for the improvement in transportation networks and alternative transportation measures to curb this menace. Also, the improvements in transportation are likely to reverse ineffective vaccination trends as evidence from some developing economies has highlighted that health workers are most interested in the achievement of vaccination coverages at the expense of the quality of the vaccines that are to be administered [43].

### 4.9. Strengths and Limitations of the Study

One of the strengths of current study is the use of quantitative and qualitative methods in answering the research questions where they were deemed appropriate. The use of census sampling in addition to validated and reliable instruments in the quantitative study can be considered as some strengths of the current study. Also, the purposive selection of participants with diverse backgrounds for inclusion in the qualitative aspect of the study as well as measures to enhance trustworthiness (credibility, conformability, dependability and transferability) contributed to the study's strength.

One of the limitations of the current study was that it was not possible to establish the relationship between knowledge, attitude, practices, and challenges on cold chain management as they were measured quantitatively or qualitatively. Thus, future studies should quantitatively measure the individual participants' knowledge, attitudes, practices, and challenges on cold chain management so that we can establish the relationships that exist between these four areas.

## 5. Conclusions

Majority of the health practitioners in the current study had a good level of knowledge and attitude towards cold chain management. While some aspects of the cold chain management practices were commendable, others needed improvement as they did not meet the required standard. Healthcare providers also encountered a number of challenges which impeded their effective management of the cold chain systems. These findings are important for effective planning and implementation of interventions to improve cold chain management. The demonstrated gaps in knowledge and attitude towards cold chain management would benefit from regular education and promotion of self-directed life-long learning among health practitioners. To militate against vaccine-induced diseases, stakeholders at the local, national, regional, and international levels should support deprived communities with the needed infrastructure and materials for the effective cold chain management. Stakeholders in cold chain management should also strengthen the monitoring activities of health facilities to ensure adherence to best practices in cold chain management. Future studies should quantitatively measure individual participants' knowledge, attitudes, practices, and challenges on cold chain management so that we can establish the relationships that exist between these components.

## Figures and Tables

**Table 1:** Sociodemographic characteristics of the participants involved in the survey (*n* = 86).

Variables	Frequency (%)
Age (years)	
21-25	7 (8.1)
26-30	48 (55.8)
31-35	2 7 (31.4)
36-40	2 (2.3)
41-45	2 (2.3)
Gender	
Female	52 (60.5)
Male	34 (39.5)
Educational qualification	
Certificate	65 (75.6)
Diploma	16 (18.6)
Bachelor's degree	5 (5.8)
Staff category	
Community health nurses	46 (53.4)
Enrolled nurses	20 (23.3)
Nurses	8 (9.3)
Midwives	8 (9.3)
Field technician	3 (3.5)
Public health officer	1 (1.2)
Subdistrict	
Nsuta	37 (43.0)
Kwamang	26 (30.2)
Oku	12 (14.0)
Birem	9 (10.5)
Asubuasu	2 (2.3)
Years of service in the Ghana Health Service	
<5	45 (52.3)
5–10	38 (44.2)
11–15	2 (2.3)
≥16 years	1 (1.2)
Years of service in cold chain management	
<5	53 (61.6)
5–10	32 (37.2)
11–15	1 (1.2)
Years of service in vaccine administration	
<5	53 (61.6)
5–10	32 (37.2)
11–15	1 (1.2)

**Table 2:** Level of knowledge and attitudes on cold chain management (*n* = 86).

Variable	Frequency (%) of categorization		
	Poor	Fair	Good
Knowledge	4 (4.7)	23 (26.7)	59 (68.6)
Attitude	9 (10.5)	19 (22.1)	58 (67.4)

Note: %: percentage.

**Table 3:** Practices on cold chain management (*n* = 12).

Variable	Frequency (%)	
	Yes (%)	No (%)
Does the facility have policies and guidelines on cold chain management practices?	1 (8.3)	11 (91.7)
Evidence of policies, procedures, and guidelines for cold chain management at this facility	1 (8.3)	11 (91.7)
Are all the staff trained to follow policies, procedures, and guidelines that ensure compliance for cold chain management?	1 (8.3)	11 (91.7)
Does the facility have a vaccine ledger book?	2 (16.7)	10 (83.3)
Does the facility have a cold chain inventory book or guide?	2 (16.7)	10 (83.3)
Are contingency plans in place with equipment?	—	12 (100)
Does the facility have an emergency power supply?	1(8.3)	11 (91.7)
Is there evidence of filling in stock cards for vaccine storage?	—	12 (100)
Is vaccine wastage managed according to policy?	—	12 (100)
Is evidence of vaccine wastage report available to make operational changes?	—	12 (100)
Is there evidence of records in case of recall/batch numbers?	8 (66.7)	4 (33.3)
Has the district trained staff on cold chain management?	10 (83.3)	2 (16.7)
District level supportive supervision and monitoring	—	12 (100)
Does the facility have a trained officer purposely in charge of cold chain management?	2 (16.7)	10 (83.3)
Does the facility have a refrigerator for storing vaccines?	11 (91.7)	1 (8.3)
Is the refrigerator technically appropriate to store vaccines (size, type, functionality, icepack compartment)?	7 (63.6)	5 (41.6)
Is the distance from the refrigerator to the wall technically appropriate?	1 (8.3)	11 (91.7)
Does the refrigerator have a lock and key?	1 (8.3)	11 (91.7)
Does the refrigerator have a functional thermometer?	1 (8.3)	11(91.7)
Functional fridge tag (if no functional thermometer)	8 (66.7)	4 (33.3)
Position of thermometer correctly placed in fridge	1 (100)	—
Absence of refrigerator (cold box fridge tag/thermometer): not applicable)	—	—
Does facility monitor temperature twice daily?	6 (50)	6 (50)
Is temperature within appropriate range? (+2°C – +8°C)	5 (41.7)	7 (58.3)
Records (30 days monthly temperature chart)	9 (75)	3 (25)
Three months reading (twice daily each day)	4 (33.3)	8 (66.7)
Level of records availability	4 (33.3)	8 (66.7)
Vaccines arranged in cold box (not applicable)	—	—
Vaccines correctly arranged in refrigerator	2 (16.7)	10 (83.3)
Diluents correctly stored in refrigerator	4 (33.3)	8 (66.7)
Are vaccines overstocked?	7 (58.3)	5 (41.7)
Space in between vaccines	1 (8.3)	11 (83.3)
Presence of food in refrigerator	—	12 (100)
Presence of water in refrigerator	—	12 (100)
Presence of medical item or biological(non-vaccine) in refrigerator	8 (66.7)	4 (33.3)
Does the facility have enough thermometer for every outreach?	—	12 (100)
Does the facility have enough functional refrigerators?	—	12 (100)
Does the facility have enough cold boxes?	5 (41.6)	7 (58.3)
Is/are the cold boxes in good condition?	4 (80)	1 (20)
Does the facility have enough vaccine carriers?	—	12 (100)
Are the vaccines in good condition?	8 (66.7)	4 (33.3)
Do all the vaccine carriers have foam pads?	15 (39.5)	23 (60.5)
Does the facility have enough thermometers or fridge tags?	—	12 (100)
Are all the available thermometers or fridge tags functional?	5 (41.7)	7 (58.3)
Does the facility have enough icepacks?	1 (8.3)	11 (91.7)
Does the facility have a deep freezer for storing icepacks?	1 (8.3)	11 (91.7)
Does the facility have enough temperature monitoring charts?	10 (83.3)	2 (16.7)
Is there enough equipment for emergency?	—	12 (100)
Does the facility have a room purposely for cold chain equipment?	5 (41.7)	7 (58.3)

## Data Availability

The datasets used and/or analyzed during the current study are available from the corresponding author upon reasonable request.

## Abbreviations

VPDs: Vaccine preventable diseases
VVM: Vaccine vial monitor.
